# Prevalence of Somatic BReast CAncer Gene (BRCA) 1 and 2 Pathogenic Variants in Portuguese Metastatic Prostate Cancer Patients

**DOI:** 10.7759/cureus.78493

**Published:** 2025-02-04

**Authors:** Tiago Barroso, Carolina Monteiro, Vanessa Patel, Lisa Gonçalves, Ana Rita Sousa, Raquel Lopes Brás, André Mansinho, Mariana Soeiro e Sá, Ana Sousa, Luís Costa

**Affiliations:** 1 Medical Oncology, Unidade Local de Saude (ULS) Santa Maria, Lisbon, PRT; 2 START Lisbon, Unidade Local de Saude (ULS) Santa Maria, Lisbon, PRT; 3 Medical Genetics, Unidade Local de Saude (ULS) Santa Maria, Lisbon, PRT

**Keywords:** brca1/2 mutations, europe, metastatic prostate cancer, parp inhibitors, portugal, prostate cancer

## Abstract

Currently, poly adenosine diphosphate ribose polymerase inhibitors are used to treat metastatic prostate cancer (mPC) patients with somatic or germline pathogenic variants in genes related to homologous recombination repair deficiency. Testing for these variants is thus advisable, as test results can have implications for systemic treatment. Of those genes, the most relevant in clinical practice are BReast CAncer gene (*BRCA*) 1and 2. Despite no published data regarding the prevalence of germline and somatic variants in mPC Portuguese patients, practitioners have long felt that the prevalence of somatic *BRCA1/2* variants in these patients is much lower than in previously studied populations. To estimate the prevalence of pathogenic *BRCA1/2* variants, we fit a Bayesian hierarchical model with data from metastatic patients subject to universal testing and data from international cohorts. All 42 patients tested were negative for somatic *BRCA1/2* pathogenic variants. This posterior estimate for the prevalence is 3.1% (95% credibility interval 0.3-10.3%), and we found a large dispersion between the prevalences of different populations. This estimate is much lower than the estimates in other published cohorts. We believe that testing recommendations should be tailored to country-specific prevalence. As such, we will continue to perform universal testing in an investigational context to decrease the uncertainty in our estimates and better establish the role of universal somatic testing in the Portuguese population.

## Introduction

Currently, guidelines from international societies such as NCCN and ESMO recommend the use of poly (ADP-ribose) polymerase (PARP) inhibitors in patients with somatic or germline pathogenic variants in genes related to homologous recombination repair (HRR) deficiency, with extensive clinical evidence behind these recommendations. PARP inhibitors have been studied for the treatment of metastatic prostate cancer as both monotherapy and combination therapy [1].

In the phase III PROfound trial [2], olaparib monotherapy has shown an increase in progression-free survival (PFS) (hazard ratio [HR] of 0.34, 95% confidence interval [CI] 0.25-0.47) benefit in patients with metastatic castration-resistant prostate cancer (mCRPC) with pathogenic somatic variants in *BRCA1*, *BRCA2*, *ATM, *and 12 other pre-specified genes (*BRIP1*, *BARD1*, *CDK12*, *CHEK1*, *CHEK2*, *FANCL*, *PALB2*, *PPP2R2A*, *RAD51B*, *RAD51C*, *RAD51D*, and *RAD54L*). Rucaparib monotherapy has also shown an objective response rate (ORR) of 43.5% (95% CI 31.0-56.7%) in mCRPC patients with pathogenic variants in *BRCA1*, *BRCA2, *and *ATM *in the phase II TRITON2 trial [3] and an increase in PFS (HR 0.61, 95% CI 0.47-0.80) in the phase III TRITON3 trial [4]. Monotherapy with niraparib has shown an ORR of 34.2% (95% 23.7-46.0%) in mCRPC patients with bi-allelic pathogenic variants in *BRCA1*, *BRCA2*, *ATM*, *FANCA*, *PALB2*, *CHEK2*, *BRIP1*, and *HDAC2 *in the phase II GALAHAD trial [5], although these results require confirmation in a phase III trial. Similarly, talazoparib has shown an ORR of 29.8% (95% CI 21.2-39.6%) in the TALAPRO-1 trial [6], an open-label phase II trial without a comparator arm.

Olaparib has been studied in combination with abiraterone compared to abiraterone alone in patients with and without HRR-deficiency biomarkers in the phase III PROpel trial [7], with a significant increase in PFS. Overall survival data are not yet conclusive, but interim results suggest a trend toward increased overall survival in the olaparib combination arm. Niraparib is also being studied in combination with abiraterone in the phase III MAGNITUDE study, which again included both patients with pathogenic gene variants causing HRR deficiency and patients without such variants. In an interim analysis, this trial has shown increased PFS (HR 0.47) in the combination arm, but overall survival data are not yet conclusive [8]. Talazoparib is being studied in combination with enzalutamide in the phase III TALAPRO-2 trial [9] in HRR-deficient metastatic castration-sensitive prostate cancer (mCRPC), and an interim analysis shows an increase in PFS (HR 0.63 95% CI 0.51-0.78). The PARP inhibitor velaparib has been tested in the phase II NCI 9012 trial [10], a trial that was negative for its primary outcome. Further combinations (including combinations with immunotherapy) are currently being tested in clinical trials [1].

Although some of the trials described above have shown benefit even in patients without HRR deficiency, with some of the drugs (in monotherapy or in combination), the benefit was larger in patients with *BRCA1 *and *BRCA2 *variants [1]. This means that biomarker testing still has a role in treatment selection. At the present date, guidelines still encourage universal testing of metastatic prostate cancer patients for HRR deficiency [11-13].

Data from several international cohorts in which patients were subject to universal testing has been published [14-19], leading to a number of estimates of the prevalence of pathogenic *BRCA1/2* variants. Due to heterogeneity in testing criteria and gene panels used, estimates of the prevalence of variants in other genes are not as easy to compare and will not be the subject of the current paper. Some of those cohorts specifically include metastatic prostate cancer patients subject to universal testing for somatic variants in *BRCA1 *and *BRCA2*. Meta-analyses have attempted to aggregate the results from such cohorts in order to produce pooled estimates, the latest of which by Valsecchi et al. [20]. The reviewed studies had prevalences from 9.4% to 16.3%, with relatively wide confidence intervals for most of the estimates. The authors reported an overall prevalence of *BRCA1 *and *BRCA2 *variants of 10.9% (95% CI 8.7-13.4%). Although aggregating several geographically separate cohorts in a meta-analysis may apparently lead to more precise estimates, one must remember that different geographical regions actually may harbor genuinely different prevalences for gene variants, both in germline testing and in somatic testing.

Portuguese oncologists (personal opinion shared among the authors, with fellow oncologists sharing the same concerns in private communication) have long felt that the yield of germline and somatic testing for metastatic prostate cancers is surprisingly low, given the prevalence estimates in the literature, which are on the order of 10% [20]. We wanted to validate or disprove this perception by estimating the prevalence of somatic pathogenic variants of *BRCA1/2* in a Portuguese population of patients with metastatic prostate cancer subject to universal testing. Because *BRCA1 *and *BRCA2 *are the most clinically important among the HRR deficiency-associated genes and because of the higher availability of data related to these two genes, we decided to focus on the prevalence of somatic variants in these genes.

Thus, our objective was to determine the prevalence of somatic *BRCA1/2* variants in Portuguese patients with metastatic prostate cancer by analyzing preliminary data from a prospective clinical trial - the Mainstreaming project.

## Materials and methods

The present paper reports original unpublished data referring to Portuguese patients included in the Mainstreaming project. We also analyzed data from international cohorts taken from the literature, with which we contrast or own data.

Portuguese cohort - the Mainstreaming project

Initially developed in England, the Mainstreaming Cancer Genetics project aimed to make cancer gene testing part of routine cancer patient care by integrating testing into the cancer patient pathway. The main objective of this project is to make genomic data available to Medical Oncologists at an earlier stage of the patient's journey, allowing for the incorporation of such data in the clinical decision process [21]. Our center adopted the recommendations of the Mainstreaming project by attempting to incorporate germline and somatic testing of HRR deficiency in the routine care of patients being treated for breast, ovarian, pancreatic, and prostate cancer. This project is a single-arm prospective trial with the goal of analyzing the impact of early genomic testing on the treatment of patients with prostate cancer, breast cancer, ovarian cancer, and pancreatic cancer.

The genetic testing for prostate cancer patients included both germline testing in blood and somatic testing in tumor tissue. The following genes were tested: *BRCA1*, *BRCA2*, *ATM*, *CHEK2*, *PALB2*, *HOXB13*, *MLH1*, *MSH2*, *MSH6, *and *PMS2*. Variants were preferably tested in tumor tissue, if available, by next-generation sequencing (NGS). In the absence of tumor tissue, peripheral blood was studied instead, also by NGS. In both cases, large exonic rearrangements (deletions and duplications) were tested by multiplex ligation-dependent probe amplification (MLPA) in peripheral blood. The Portuguese founder variant in *BRCA2* (c.156_157insAlu) was specifically tested for in peripheral blood. The techniques used were MLPA and/or polymerase chain reaction and agarose gel electrophoresis. In case of a positive result (pathogenic/likely pathogenic variants or variants of unknown significance), the patients were referred to a Medical Genetics appointment for genetic counseling of the patient and family members.

In the setting of localized disease, patients are eligible for testing if either 1) the tumor has intraductal, ductal, or cribiform histology or 2) the patient has high-risk features (tumor staging ≥ T3, Gleason score ≥ 8, or prostate-specific antigen [PSA] ≥ 20 ng/mL) and a next-of-kin diagnosed with prostate cancer before the age of 60 or breast cancer before the age of 50. By contrast, all patients with metastatic disease are eligible for testing, as long as they are eligible for systemic treatment according to the attending Oncologist.

We present the data from the subset of the metastatic patients. Thus, we included in our cohort all metastatic patients, independent of age, who were subject to somatic testing for genes related to homologous recombination deficiency and for whom the test results were available between January 2018 and November 2024.

International cohorts

The international cohorts [14-19] analyzed in this paper are the ones reviewed in the already published 2023 meta-analysis [20]. To the best of our knowledge, this is the latest meta-analysis that has looked at the prevalence of the *BRCA1* and *BRCA2* variants in cohorts of prostate cancer patients submitted to universal testing. The original papers were reviewed to collect the number of total and positive patients and to review the patient’s characteristics.

Bayesian hierarchical model and visualization

We have built a simple Bayesian hierarchical binomial model similar to the one described implemented by Carpenter et al. [22]. Instead of the more commonly used frequentist method, we chose to use a Bayesian approach as it allows us to use of hierarchical models in a natural way.

Because of different environmental exposures, founder effects and lack of mixing of geographically separate populations, we expect the prevalence of BRCA1/2 mutations to be different in different geographical regions. That is, each individual cohort will have a true prevalence $\theta_i$. These prevalences should cluster around a worldwide mean value. We can thus model the distribution of these prevalences as a $\text{Beta\_Proportion}(\mu, \kappa)$ distribution with mean ($\mu$) and dispersion ($\kappa$). The $\text{Beta\_Proportion}(\mu, \kappa)$ distribution is an alternate parametrization of the Beta distribution, such that $\text{Beta\_Proportion}(\mu, \kappa)$ is equivalent to $\text{Beta}(\mu\kappa, (1 - \mu)\kappa)$. Informally, we exploit both the differences and similarities between populations around the world in a mathematicaly sound way in order to refine the estimate for the true prevalence $\theta_i$ in each population. This refinement is more important for smaller populations.

For each population with prevalence $\theta_i$ and $N_i$, the number of positive patients $P_i$ will follow a binomial distribution with parameters $N_i$ and $\theta_i$. The common dependence of $\theta_i$ on $\mu$ and $\kappa$ is what makes the model hierarchical. With this model, the prevalences $\theta_i$ will cluster around the mean $\mu$. The dispersion $\kappa$ is a measurement of how far apart those prevalences will be. Larger values of $\kappa$ cause population prevalences to be very different from each other, while smaller values of $\kappa$ will cause population prevalences to be closer to the mean. The hierarchical approach may lead to better estimates for cohorts with fewer patients. It is also common to define unadjusted prevalences $\rho_i$, which are not dependent on $\mu$ and $\kappa$. This will allow us to see how much the estimated prevalence values are influenced by the other cohorts.

Formally, we can define the model as:

$\theta_i \sim \text{Beta\_Proportion}(\mu, \kappa)$ for all $i$

$P_i \sim \text{Binomial}(N_i, \theta_i )$ for all $i$

$\mu \sim \text{Beta}(1, 1)$

$\kappa \sim \text{Gamma}(0.1, 1)$

For the unadjusted prevalences, we define:

$\rho_i \sim \text{Beta}(1, 1)$ for all $i$

$P_i \sim \text{Binomial}(N_i , \rho_i )$ for all $i$

The graphical representation in Figure 1 can help understand how the model parameters relate to each other and how the model exploits the relations between populations in order to refine the population estimates.

**Figure 1:** Graphical representation of the Bayesian hierarchical model Bayesian hierarchical models aim to take advantage of clustering of data on various levels. They can often be represented graphically, and graphical representations can help comprehension. In the current model, we can think of three conceptual levels in the hierarchy. On the top level, we have an aggregate of populations containing parameters, which will influence the population prevalence. On the middle level, we have the individual populations. In this model, populations are different from each other (each has its own prevalence *θ_i_*, total number of patients *N_i_*, and total number of positive patients *P_i_*). However, they are also related to each other through the mean (*μ*) and dispersion (*κ*) parameters of the top level, as the prevalence *θ_i_* depends on both *μ* and *κ*. On the bottom level, we can think about individual patient data. Patients are naturally different from each other, but at the same time they are related to one another through the parameters of their respective populations. Although for clarity we represent the individual patients as a level of the hierarchy, our model does not use individual patient data. Please refer to the text for a more detailed explanation of the model parameters.

The model was implemented in the Stan programming language [23] together with CmdStanPy [24]. We fit the models to the available data and stimulated the posterior distribution of the model parameters. The full Stan code that implements the model above is a straightforward translation of the mathematical model and can be found in the Appendix.

Data processing, visualization, and reporting of results

Data processing was done in the Python programming language [25], with the Pandas [26] and NumPy [27] packages. Posterior distributions were plotted with a custom Python program using the Matplotlib package. Whenever kernel density estimations of distributions were plotted, we used the ArViz package [28]. In the text and tables, each estimate was reported as a 95% credible interval (CdI) centered around the median.

## Results

We identified 42 patients with metastatic prostate cancer who underwent somatic testing according to the inclusion criteria. Although our testing protocol allowed for biopsy of both the primary tumor and metastasis, all biopsies were from the primary tumor. The median age was 72 years (interquartile range: 66-79). The age of the patients in the other cohorts is shown in Table 1. In our cohort (referred to in the tables as Barroso et al., 2024), all somatic tests for *BRCA1/2* variants were negative (zero positive patients out of 42). One patient had a likely pathogenic *CHEK*2 somatic variant. The adjusted median of the posterior adjusted prevalence was 3.1% (95% CdI 0.3-10.3%). Regarding the Beta_Proportion distribution parameters, the posterior median of the median prevalence ($\mu$) was 11.6% (95% CdI 6.8-20.1%) and dispersion ($\kappa$) was 19.1 (95% CdI 4.79-54.15). In Figure 2, we show the full posterior probability distributions for the model parameters, including the adjusted and unadjusted prevalences for the seven cohorts. The number of total and positive patients of the other 6 cohorts, the age range, and the estimated adjusted and unadjusted prevalences (median and 95% CdI) are shown in Table 2.

**Table 1:** Cohort characteristics for the analyzed cohorts Cohort characteristics for the analyzed cohorts. The first six cohorts (from 2015 to 2022) are those analyzed in the 2023 meta-analysis, and only the last cohort (Barroso et al., 2024) contains original data. Ages and age ranges are displayed in years and are rounded to the nearest integer.

	Age - mean (IQR)	Total no. of patients	No. of positive patients
Robinson et al., 2015 [14]	Not reported	150	19
Mateo et al., 2015 [15]	67.5 (41–80)	49	8
Mota et al., 2020 [16]	68 (63–74)	64	6
Tukachinsky et al., 2021 [17]	71 (38–89)	837	71
Martinez Chanza et al., 2021 [19]	65 (44–88)	141	14
Uemura et al., 2022 [18]	73 (52–90)	143	19
Barroso et al., 2024	72 (66–79)	42	0

**Figure 2:** Posterior estimates of parameter values for the model (A, B) Parameters - mean $\mu$ and dispersion $\kappa$ - of the Beta_Proportional distribution, which generates the individual cohort prevalences. The black horizontal lines correspond to the 95% CdI and the dot in the middle corresponds to the median of the posterior distribution. (C-I) Posterior probability estimates of the adjusted and unadjusted prevalence of somatic BRCA1/2 variants in individual cohorts. Plots C-H correspond to the populations already studied in the 2023 meta-analysis, while plot I corresponds to the cohort from our center (the only one that brings data original to this paper). In plots C-H, the semi-transparent blue distribution corresponds to the unadjusted prevalences $(\rho_1, \dots, \rho_7)$, while the semi-transparent orange distribution corresponds to the adjusted prevalences $(\theta_1, \dots, \theta_7)$. The black line under the distribution corresponds to the 95% CdI of the adjusted prevalence, and the black dot in the middle corresponds to the median of the posterior distribution of the adjusted prevalence. The intervals for the adjusted prevalences are not shown. In the top right corner of plots C-I, we show the absolute difference between the median of the posterior of the adjusted prevalence and the median of the posterior of the unadjusted prevalence. The x-axes of plots A and C-I have the same scale, so that parameter values can be directly compared. Plot B (dispersion, $\kappa$) has a different scale, as $\kappa$ cannot be meaningfully compared to population prevalences.

**Table 2:** Adjusted and unadjusted estimates for BRCA1 or BRCA2 variant prevalence for each cohort See the text for further details regarding the model fitting and the meaning of the adjusted prevalences. The first six cohorts (from 2015 to 2022) are those analyzed in the 2023 meta-analysis, and only the last cohort (Barroso et al., 2024) contains original data. Although data from the first six cohorts has been previously published, the Bayesian estimates for the prevalence are new. The *r_hat* values very close to 1.0 show that all model chains converge correctly in the simulations.

	Adjusted prevalence $\theta_i$			Unadjusted prevalence $\rho_i$		
	Median	95% CdI	r _hat	Median	95% CdI	r _hat
Robinson et al., 2015 [14]	12.4%	8.0-17.9%	1.000	13.0%	8.2-19.0%	1.000
Mateo et al., 2015 [15]	14.6%	7.5-24.8%	1.000	17.2%	8.6-29.2%	1.000
Mota et al., 2020 [16]	9.5%	4.5-17.2%	1.000	10.2%	4.4-19.0%	1.000
Tukachinsky et al., 2021 [17]	8.5%	6.8-10.5%	1.000	8.5%	6.8-10.6%	1.000
Martinez Chanza et al., 2021 [19]	10.0%	6.0-15.2%	1.000	10.3%	6.0-16.1%	1.000
Uemura et al., 2022 [18]	12.9%	8.3-18.7%	1.000	13.7%	8.7-19.9%	1.000
Barroso et al., 2024	3.1%	0.3-10.3%	1.000	1.7%	0.2-8.2%	1.000

## Discussion

We have estimated that the prevalence of pathogenic *BRCA1/2* variants in Portuguese patients with metastatic prostate cancer subject to universal testing is 3.1% (95% credibility interval 0.3-10.3%). However, in our cohort, despite the long duration of data collection and the fact that our center has a relatively high volume of metastatic prostate cancer patients, the total number of patients with somatic testing was low. This has two main causes. First, in the first years of implementation of the project, due to a lower level of standardization of medical care, not all prescribers complied strictly with the testing protocol. Second, when a primary tumor sample was unavailable due to inability to locate the sample in the center where it was collected or when sample characteristics (samples that were too old or those with a very low number of neoplastic cells) did not allow for comprehensive genetic testing in tissue, somatic testing results are not available, as only germline testing could be correctly performed. Due to the high prevalence of bone-only disease in prostate cancer patients and due to the difficulty of genetic testing in biopsies from bone disease, all tissue was gathered from the primary tumor.

The main limitation in our estimate of the true *BRCA1/2 *variant prevalence is the relatively low number of patients with somatic testing, which leads to an uncertain estimate: median 3.1% (95% CdI 0.3-10.3%). As we continue to perform universal somatic testing in metastatic patients, we expect to gather more data and decrease the uncertainty of our prevalence estimates.

Both the adjusted and the unadjusted prevalences of *BRCA1/2* variants were much lower in the Portuguese cohort than in the other six analyzed cohorts. The use of a Bayesian hierarchical model is a strength, as it helps reduce uncertainty and improve accuracy in small populations such as ours, when compared to the use of unadjusted prevalences. For these cohorts, however, we found out that adjusted and unadjusted estimates are similar (Table 2). Still, low sample sizes in both the Portuguese cohort (N = 42) and in other cohorts leads to prevalence estimates which are quite uncertain, with wide confidence intervals. The posterior median for the mean population prevalence is 11.6% (CdI 6.8-20.1%), which is much higher than the 3.1%, the median prevalence in the Portuguese cohort. The posterior median for the dispersion is 19.1 (95% CdI 4.79-54.1). This high dispersion value supports the fact that the *BRCA1/2* variant prevalence is heterogeneous among populations and that the low prevalence in the Portuguese population may reflect a truly low prevalence instead of being just a statistical artifact from the relatively low sample size. Unfortunately, the low size of some of the populations and the low number of cohorts (only seven cohorts, including ours) makes it hard to estimate the true value for the dispersion.

It is not clear what is the cause behind the large prevalence differences between the Portuguese population and the international populations. While one might suspect methodological effects causing some of the prevalence estimates to be biased, all populations (including all own) report data from non-selected patients subject to universal testing. Median age is similar among the seven cohorts (Table 1), which further supports the idea that patient choice is relatively unbiased. This supports the existence of a real biological differences between populations. The difference between the Portuguese cohort and the other cohorts could be due to founder effects, although our data can neither confirm or refute this hypothesis. Answering these questions will probably require more advanced genetic tools than the ones we have employed here.

The main limitation of our study was the low sample size. With only 42 tested patients and a relatively wide credibility interval, our data can not currently be used to recommend country-specific changes in testing guidelines. In the future, we will continue to test patients for germline and somatic markers HRR deficiency in an investigational context in order to increase the precision of our prevalence estimates. This will help better establish the role of universal somatic testing for *BRCA1 *and *BRCA2* pathogenic variants in clinical practice in Portuguese patients.

## Conclusions

We have, for the first time, published an estimate of the prevalence of *BRCA1/2* pathogenic variants in Portuguese patients with metastatic prostate cancer. The prevalence in our population was estimated as 3.1% (95% CdI 0.3-10.3%), lower than in previously published cohorts from other countries. While from a medical point of view, testing of available tumor samples for *BRCA1/2* and other HRR deficiency-associated genes is free from risk to the patient (barring the rare event of an error during sequencing, which may lead to suboptimal systemic treatment), from a pharmaco-economical point of view, universal testing in the absence of clinical risk factors is harder to justify if the baseline prevalence is low. Policy recommendations should consider both the benefits of testing and the cost of sequencing a large number of patients. In the case of *BRCA1 *and *BRCA2 *genetic variants, we believe that guidelines should acknowledge the fact that universal testing should be guided by the local prevalence of HRR deficiency-associated variants.

## Appendices

Stan code

The following stan code implements the model described in the text:

data {    // Nr. of studies    int<lower=0> N_studies;    // Number of total patients per study    array[N_studies] int totals;    // Number of positive patients per study    array[N_studies] int positives; } parameters {    // Parameters of the beta_proportion distribution    real<lower=0.001, upper=0.999> mu;    real<lower=0.001> kappa;    // Study-level probabilities    vector<lower=0.001, upper=0.999>[N_studies] unadjusted_theta;    vector<lower=0.001, upper=0.999>[N_studies] adjusted_theta; } model {    // Hyperprior    mu ~ beta(1, 1);    kappa ~ gamma(1.0, 0.1);    unadjusted_theta ~ beta(1, 1);    adjusted_theta ~ beta_proportion(mu, kappa);    positives ~ binomial(totals, adjusted_theta);    positives ~ binomial(totals, unadjusted_theta); }
